# Nutritive value of faba bean (*Vicia faba* L.) as a feedstuff resource in livestock nutrition: A review

**DOI:** 10.1002/fsn3.2342

**Published:** 2021-07-22

**Authors:** Zhu Meng, Qingqing Liu, Yan Zhang, Jiahong Chen, Zhipeng Sun, Chunhuan Ren, Zijun Zhang, Xiao Cheng, Yafeng Huang

**Affiliations:** ^1^ Department of Animal Science and Technology Anhui Agricultural University Hefei China; ^2^ Center of Agriculture Technology Cooperation and Promotion of Dingyuan County Chuzhou China

**Keywords:** animal feeding, antinutritional factors, faba bean, nutrition value, performance

## Abstract

The review evaluates faba bean (*Vicia faba* L.; FB) seeds relative to their nutritional composition, their content of antinutritional factors, and their impact on animal performance. The literature indicates that FB plant is a cool‐season, annual grain legume that grows the best in cool and humid conditions. Its seeds are rich in protein, energy, and mineral compounds and have particularly high unsaturated fatty acid levels. However, FB seeds also contain various proportions of antinutritional factors (ANFs) that can interfere with nutrient utilization in nonruminants. The various processing methods are efficient in either reducing or inactivating the ANFs of FB seeds, with extrusion treatment offering the most effective method of improving apparent nutrient and energy digestibility of nonruminants. In vivo studies on ruminants, pigs, poultry, and fishes reveal that FB seeds have the potential to be used as a substitute for soybean meal and/or cereal seeds in livestock diets in order to support milk, meat, and/or egg production.

## Abstract 2

Faba bean plant is a cool‐season, annual grain legume that grows the best in cool and humid conditions. Its seeds are rich in protein, energy, and mineral compounds and have particularly high unsaturated fatty acid levels. Its seeds have the potential to be used as a substitute for soybean meal and/or cereal seeds in livestock diets in order to support milk, meat, and/or egg production.

## 1 INTRODUCTION

The faba bean (FB) (*Vicia faba* L.; Fabales: Fabaceae) is a cool‐season, annual grain legume crop, traditionally used as a significant and cheap plant protein source for human and livestock diets (Elsheikh et al., 1999; Gu et al., 2020). Although the V. *faba* plant originated in the Middle East during prehistoric times (Multari et al., 2015), it is now cultivated worldwide (Prabhu & Rajeswari, 2018) and ranked as the third most important grain legume (Gu et al., 2020). Globally, the production area of the FB is 2,511,813 ha, equating to a crop production yield of 4,923,154 tonnes/year and an average annual yield of 1,960 kg/ha (FAO, 2018). China is the leading FB producer with 36.7% of the global output, followed by Ethiopia (20.1%), the United Kingdom (8.2%), and Australia (7.7%) (FAO, 2018).

The FB plant has the ability to suitability for cultivation in any climate (Singh et al., 2013), where soybean is poorly suited to cool climates (Duc et al., 2015), or where perennial forage legumes perform poorly under high‐altitude conditions with a short growing season (<100 days) (Huang et al., 2019; Stoddard & Hämäläinen, 2011). The cool and moist conditions are regarded as the best growth conditions for the FB plant (Duc et al., 2015). Moreover, FB can be cultivated across a range of soil environment types, especially in areas with the poorest soil types in which barley and wheat perform poorly (Castanon et al., 1990). However, fine‐textured soils and soils with pH levels >7 are considered to provide the ideal soil conditions for cultivating FB (Etemadi et al., 2019; Köpke & Nemecek, 2010). Additionally, FB plants stand out for their N fixation efficiency, which is the highest among the cool‐season legumes (Álvarez‐Iglesias et al., 2018; Olson & Bowness, 2016), and can facilitate the reduction in the use of commercial N fertilizers, providing ecosystem services that contribute to sustainable agriculture (Khazaei et al., 2019).

Although FB seeds play an important role as a source of nutrition in human diets (Etemadi et al., 2018), they also provide the livestock industry with an alternative protein and energy feedstuff source to offset feed costs and ensure a stable feed supply for livestock (Etemadi et al., 2019; Smith et al., 2013). This review elucidates the nutrient profile of FB seeds and their use in animal diets to promote their use in livestock diets.

## 2 NUTRITIONAL COMPOSITION OF THE FABA BEAN

### 2.1 Proximate nutrients

The proximate nutritional content of FB sees is given in Table 1. FB seeds contain 210–341 g/kg dry matter (DM), with globulins (61.35% crude protein [CP]) and albumin (20.02% CP) being the major components (Gasim et al., 2015). The total carbohydrate content of FB seeds ranges from 457 to 701 g/kg DM, with starch, total sugars, and fiber as the major carbohydrate components (Khan et al., 2015; Morales et al., 2008). In addition, FB seeds are also good sources of dietary minerals (Cazzato et al., 2014), notably potassium, phosphorus, iron, and zinc, while iron and zinc are essential for the sustenance and optimal physiological function of both humans and livestock (Bailey et al., 2015). The gross energy and metabolizable energy (ME) contents of FB seeds, which range from 14.69 to 19.70 MJ/kg DM and from 11.30 to 13.80 MJ/kg DM, respectively. The chemical composition content of FB seeds is highly dependent on the genotypes/cultivars and environmental conditions, as well as agricultural management practices (Ivarsson & Neil, 2018; Micek et al., 2015; Pelagalli et al., 2020; Skylas et al., 2019). Compared with general grains such as rice, corn and wheat, FB seeds contain higher CP, dietary fiber, potassium, iron, and folic acid contents (Howard et al., 2018; Gu et al., 2020).

**TABLE 1:** The proximate nutritional content (g/kg dry matter, unless otherwise stated) of faba bean seeds summarized from several references^a^

Nutrients	*n* ^b^	Mean	Minimum	Maximum	*SD*
Dry matter (g/kg)	23	893.92	859.5	960.05	23.22
Organic matter	6	944.55	854.5	965.8	40.33
Ash	18	40.5	28.7	73	11.21
Crude protein	30	282.22	210	340.63	29.37
Ether extract	22	17.62	8.4	41	7.68
Crude fiber	13	97.21	15	224	43.77
Neutral detergent fiber	14	220.6	119	426	83.83
Acid detergent fiber	10	115.78	102.6	134.7	10.76
Acid detergent lignin	5	25.12	19.1	40	7.59
Total carbohydrates	3	565.27	457	701	101.49
Nitrogen‐free extract	4	488.33	381	619	97.46
Starch	10	360.1	300.74	417	40.78
Sugar	1	42.8	40	45.6	2.8
Potassium	2	9.76	7.53	12	2.24
Phosphorus	5	3.74	0.69	5.62	1.87
Calcium	5	2.24	0.37	3.9	1.39
Magnesium	3	0.93	0.08	1.4	0.6
Chlorine	1	1	1	1	0
Sodium	1	0.5	0.5	0.5	0
Iron (mg/kg DM)	2	116.65	81.5	151.8	35.15
Zinc (mg/kg DM)	2	52	40	64	12
Manganese (mg/kg DM)	2	26.4	24.8	28	1.6
Copper (mg/kg DM)	1	24.9	24.9	24.9	0
Gross energy (MJ/kg DM)	7	17.85	14.69	19.7	1.69
Metabolizable energy (MJ/kg DM)	3	12.63	11.3	13.8	1.03
Digestible energy (MJ/kg DM)	2	14.6	14.19	15	0.41

Abbreviation: *SD*, standard deviation.

^a^ Supporting literature: (Aguilera et al., 1992; Azaza et al., 2009; Barłóg et al., 2019; Benchaar et al., 1994; Berger et al., 1999; Cherif et al., 2018; Cucci et al., 2019; Dixon & Hosking, 1992; Elsheikh et al., 1999; Ferruzzi et al., 2009; Gous, 2011; Hadjipanaiotou et al., 1985; Hejdysz et al., 2016; Ivarsson & Neil, 2018; Koivunen, Tuunainen, Rossow, et al., 2014; Kumar et al., 2015; Lamminen et al., 2019; Masoero et al., 2005; Micek et al., 2015; Morales et al., 2008; Moujahed et al., 2020; Rotger et al., 2006; Rubio et al., 1992; Skylas et al., 2019; Smith et al., 2013; Soltanzadeh et al., 2017; Vaga et al., 2017; Zagorakis et al., 2015).

^b^ Number of supporting literature.

### 2.2 Fatty acids and amino acids

The FB seeds contain 38.70 g/kg of total lipids (Akpinar et al., 2001). The major unsaturated fatty acids in FB seeds are the oleic (56.5 g/kg), palmitoleic (37.3 g/kg), and linoleic (36.4 g/kg) acids, while the palmitic (67.3 g/kg) and stearic (34.9 g/kg) acids constitute the major saturated fatty acid components of FB (Angell et al., 2016). These results indicate that combined with the high CP content, the unsaturated fatty acid level of FB seeds makes them a low‐cost, vegetable protein source for both humans and livestock.

The total amino acid (TAA) content of FB seeds ranges from 217.4 to 322.7 g/kg DM (Table 2). Of the amino acids, essential amino acids (EAAs) account for 132.5 g/kg DM (arginine 25.3 g/kg DM, leucine 20.4 g/kg DM, and lysine 17.9 g/kg DM), with a higher EAA/TAA ratio than soybean [*Glycine max* (Linn.) Merr.] meal (SBM) (mean EAA)/TAA = 52.0% and 46.0%, respectively) (Angell et al., 2016), thereby indicating that FB seeds contain protein of a higher quality than SBM. For nonessential amino acids (NEAA), FB seeds constitute 125.4 g/kg DM (glutamic acid 47.9 g/kg DM and aspartic acid 30.7 g/kg DM); however, there may be some differences in the sequence and general structure of amino acids (El Fiel et al., 2002). FB seeds, with their higher levels of lysine and arginine, could be mixed with cereals that would supplement some of the EAA compounds that FB lacks, thereby achieving a more balanced and desirable amino acid profile (Kumar et al., 2015; Skylas et al., 2019).

**TABLE 2:** Amino acid composition (g/kg dry matter) of faba bean seed summarized from several references^a^

Constituent	*n* ^b^	Mean	Minimum	Maximum	*SD*
Crude protein	7	300.9	272.6	340.6	22
Essential amino acid					
Lysine	7	16.3	6.7	20.8	4.2
Threonine	7	9.3	3.5	12.9	2.7
Methionine	7	2	0.9	2.9	0.6
Cystine	7	2.8	1	4.1	1.1
Isoleucine	7	9.8	3.9	11.7	2.6
Valine	7	11.2	4.4	13.6	3
Leucine	7	18.6	7.1	25.4	5.3
Phenylalanine	7	10.6	4.1	12.7	2.7
Histidine	7	7.2	2.8	8.9	1.9
Arginine	7	22.5	9.8	27.8	5.6
Glycine	7	10.9	4	14.7	3.1
Non‐essential amino acid					
Tyrosine	7	8	2.9	10	2.3
Alanine	7	10.7	3.9	15.1	3.2
Aspartic acid	7	26.9	10.2	38.6	8.1
Glutamic acid	7	42.8	14.9	57.5	12.4
Serine	7	12.4	4.4	18.4	3.9
Proline	7	11.7	4	18.7	4.1

Abbreviation: *SD*, standard deviation.

^a^ Supporting literature: (Aguilera et al., 1992; Barłóg et al., 2019; Biesek et al., 2020; Hejdysz et al., 2016; Ivarsson & Neil, 2018; Koivunen, Tuunainen, Rossow, et al., 2014; Koivunen et al., 2016).

^b^ Number of supporting literature.

Overall, FB seeds, as relatively complete feed, provide a rich source of protein, carbohydrates, fats, and minerals, with potential for incorporation into animal diets.

## 3 FACTORS IMPAIRING THE UTILIZATION OF FABA BEAN IN LIVESTOCK FEEDSTUFF

Despite being rich in protein, carbohydrates, fats, and minerals, FB seeds contain a variety of antinutritional factors (ANFs), such as total phenolics, tannins, and trypsin inhibitor activity (TIA) (Table 3) (Ferruzzi et al., 2009; Hejdysz et al., 2016). These ANFs adversely affect the feed palatability as well as the bioavailability of protein and energy, thereby potentially interfering with certain animal performance indicators such as growth and egg production (Barłóg et al., 2019; Kowalczyk et al., 2020; Multari et al., 2015). For raw FB seeds, ANFs constitute 8.50–28.48 g/kg of total phenolics, 3.80–14.50 g/kg of tannins, 1.61–10.11 g/kg of phytic acid, 16.90–24.02 g/kg of verbascose, 7.60–18.70 g/kg of stachyose, 2.00–4.50 g/kg of raffinose, and 0.60–1.50 g/kg of TIA, depending on the genotype/cultivar, environmental conditions, growing season, seed maturity stage, and agronomic practices implemented (Cucci et al., 2019; Ivarsson & Neil, 2018; Kowalczyk et al., 2020; Oomah et al., 2011). The variation in ANFs in FB seeds may limit their use in feed formulations of animal diets.

**TABLE 3:** Antinutritional compounds (g/kg, unless otherwise stated) of faba bean seed summarized from several references^a^

Constituent	*n* ^b^	Mean	Minimum	Maximum	*SD*
Total phenolics	3	17.59	10.7	28.48	7.79
Tannins	6	7.38	0.06	14.5	4.72
Vicine	5	5.95	0.99	12.38	3.81
Phytic acid	4	9.24	1.7	21.25	7.59
Convicine	5	2.72	1.35	3.88	0.81
Poliphenols	1	2.49	–	–	–
Trypsin inhibitor activity	4	0.9	0.6	1.5	0.36
Daidzein (ppm)	1	0.1	–	–	–
Oligosaccharides					
Verbascose	2	3	25.79	16.9	36.44
Stachyose	2	3	13.44	7.6	18.7
Raffinose	3	4	3.26	2	4.5

Abbreviation: *SD*, standard deviation.

^a^ Supporting literature: (Abusin et al., 2009; Berger et al., 1999; Biesek et al., 2020; Cucci et al., 2019; Drażbo et al., 2018; Elsheikh et al., 1999; Ferruzzi et al., 2009; Gdala & Buraczewska, 1997; Hejdysz et al., 2016; Khalil & Mansour, 1995; Landry et al., 2016; Masoero et al., 2005; Oomah et al., 2011; Purves et al., 2017; Skylas et al., 2019; Smith et al., 2013; Van der Poel et al., 1991).

^b^ Number of supporting literature.

Relative to other legumes, such as soybeans and peas (*Pisum sativum* L.), FB seeds contain similar amounts of tannins and polyphenols, but relatively less TIA, genistein, and daidzein content (Berger et al., 1999), which indicates that FB seeds may less impair the nonruminant nutrition status. However, in ruminants, the ANFs in FB seeds and other seed legumes do not have a substantive effect on nutrient absorption in the small intestine of ruminants because the ANFs might be inactivated after 12–24 hr of in vitro incubation with rumen liquor (Holmes et al., 1993). In fact, tannins in the ANFs might even be beneficial in terms of protein absorption in the small intestine, since high tannin levels in the diet can form stable complexes which protect proteins from rumen microbial degradation (Mohamaden et al., 2020). As indicated in the literature, high inclusion rates of raw FB seeds in diets do not negatively affect the growth performance of male lambs (Bonanno et al., 2012; Lanza et al., 1999).

## 4 BIOLOGICAL EVALUATION OF THE FABA BEAN

The biological evaluation of FB protein is of critical importance not only in terms of reflecting its potential as an animal feed, but also because chemical analyses do not always reflect the bioavailability and utilization of nutrients in animals (Huang et al., 2019). The intestinal availability of rumen undegradable protein (IARUP), protein efficiency ratio (PER), rumen available energy (PDIE), and rumen available nitrogen (PDIN) are the critical parameters for determining the biological value of grain legumes (Eckert et al., 2019; Micek et al., 2015). In ruminants, the IARUP and PDIN from raw FB seeds ranged from 0.662 to 0.777 (Benchaar et al., 1994; Espinosa et al., 2020) and from 0.191 to 0.197 (Micek et al., 2015), respectively, while PER ranged from 2.40 to 2.86 for nonruminants (Eckert et al., 2019; Khalil & Mansour, 1995). The BV and PDIE of raw FB seeds were 0.630 and 0.114, respectively (Eckert et al., 2019; Micek et al., 2015).

### 4.1 In vitro digestibility

A summary of the in vitro digestibility of FB seeds is shown in Table 4. The in vitro organic matter (OM) and CP digestibility of raw FB seeds ranged from 0.725 to 0.914 (Ferruzzi et al., 2009; Ivarsson & Neil, 2018) and from 0.646 to 0.955, respectively (Chandra‐Hioe et al., 2016; Ivarsson & Neil, 2018; Khalil & Mansour, 1995). The in vitro DM and neutral detergent fiber (NDF) digestibility of raw FB seeds were 0.735 and 0.518, respectively (Ferruzzi et al., 2009; Ivarsson & Neil, 2018). Overall, FB seeds have a considerable variation in terms of the in vitro digestibility of their nutrients, which largely depends on the cultivar type, the environmental conditions the crops grown in, and the agronomic practices implemented (Abusin et al., 2009; Buckley et al., 1983; Ivarsson & Neil, 2018; Stone et al., 2019).

**TABLE 4:** The in vitro nutrient digestibility of the faba bean (FB) seeds summarized from several references

Authors	Feedstuff	In vitro digestibility			
		DM	OM	CP	NDF
Van der Poel et al. (1991)	Raw FB seed	–	–	0.935	–
	Extruded FB seed	–	–	0.948	–
Khalil and Mansour (1995)	Raw FB seed	–	–	0.646	–
	Cooked FB seed	–	–	0.712	–
	Autoclaved FB seed	–	–	0.737	–
	Germinated FB seed	–	–	0.722	–
Elsheikh et al. (1999)	Raw FB seed	–	–	0.733	–
Ferruzzi et al. (2009)	Raw FB seed	–	0.914	–	0.518
	Dehulled FB seed	–	0.993	–	0.903
	Flaked FB seed	–	0.925	–	0.554
	Cooked FB seed	–	0.895	–	0.487
	Germinated FB seed	–	0.904	–	0.391
Chandra‐Hioe et al. (2016)	Raw FB seed	–	–	0.755	–
Ivarsson and Neil (2018)	Raw FB seed	0.735	0.725	0.955	–
Stone et al. (2019)	Raw FB seed	–	–	0.769	–

Abbreviations: CP, crude protein; DM, dry matter; NDF, neutral detergent fiber; OM, organic matter.

### 4.2 Ruminal degradability, in vivo digestibility in ruminants, and fermentation characteristics

The ruminal degradability of the CP of raw FB is 0.794 (on a DM basis) and 0.810 in cows and heifers (Table 5), respectively (Cherif et al., 2018; Rotger et al., 2006), and as high as 0.880 in rams (Zagorakis et al., 2015). In addition, the ruminal CP degradability of raw FB seeds has been reported to be 0.892 g/kg and 0.857 g/kg at two outflow rates, respectively, in mature wethers (Aguilera et al., 1992). In sheep, the ruminal CP degradability increased with increased dietary FB seed proportion and decreased with increased size of grinding particles from coarse (2 mm) to fine (1 mm) (Dixon & Hosking, 1992). The ruminal DM and CP degradability of raw FB seeds was largely variable, perhaps depending on the cultivar type, environmental conditions, livestock species, basal diet, rumen outflow rate, and ground particle size.

**TABLE 5:** Effective degradability of faba bean (FB) seeds summarized from several references and different animal species

Authors	Animal	Feedstuff	Outflow rate (/hr)	Effective degradability	
				DM	CP
Aguilera et al. (1992)	Mature wethers	Raw FB seed	0.015	0.808	0.892
			0.022	0.761	0.857
		AutoclavedFB seed	0.015	0.697	0.769
			0.022	0.621	0.703
Rotger et al. (2006)	Heifers	Raw FB seed	–	–	0.810
Morales et al. (2008)	Dairy goats	Raw FB seed	0.030	–	0.862
Zagorakis et al. (2015)	Rams	Raw FB seed	0.020	0.771	0.880
Cherif et al. (2018)	Cows	Raw FB seed	–	0.711	0.794
		Rolled FB seed	–	0.516	0.532

Abbreviations: CP, crude protein; DM, dry matter.

In ram diets containing FB seeds (162 g/kg), the apparent digestibility of DM, OM, and CP was somewhat lower than that of the SBM control diet (156 g/kg; Table 6), while the apparent digestibility of DM, OM, and CP in raw FB diets was similar to that of the SBM control diet (Zagorakis et al., 2015). On the contrary, in cows, the apparent digestibility of DM, OM, CP, NDF, starch, and energy, as well as N retention were generally unaffected by increasing levels of raw FB seeds (Puhakka et al., 2016). In addition, Cherif et al. (2018) reported that similarities in the apparent digestibility of certain dietary components (i.e., DM, OM, CP, NDF, acid detergent fiber [ADF], starch, and energy) between diets of lactating cows that were fed with raw FB seeds (171 g/kg DM) and those fed with an SBM diets (92 g/kg DM). Overall, the apparent DM, OM, and CP digestibility in the raw FB seed diets was higher in wethers than in rams and lactating cows (Cherif et al., 2018; Hadjipanaiotou et al., 1985; Zagorakis et al., 2015).

**TABLE 6:** Nutrient and energy digestibility (g/kg), and N retention (g/day) of faba bean (FB; g/kg DM, unless otherwise stated) seed summarized from several references and different ruminant species

Authors	Animal	Feedstuff	FB level	Nutrient digestibility							ED	N retention
				DM	OM	CP	EE	NDF	ADF	Starch		
Hadjipanaiotou et al. (1985)	Wethers	Raw FB seed (g/kg)	288	800	820	810	–	–	–	–	780	–
Zagorakis et al. (2015)	Rams	Raw FB seed (g/kg)	0	709	736	721	767	531	417	–	–	–
			162	687	716	690	753	520	383	–	–	–
Puhakka et al. (2016)	Cows	Raw FB seed	0	728	742	682	–	624	–	948	–	163
			75.1	730	746	665	–	647	–	951	–	157
			150	726	741	681	–	608	–	954	–	151
			175	722	738	693	–	632	–	931	–	160
			350	738	753	719	–	607	–	961	–	146
Cherif et al. (2018)	Lactating cows	Raw FB seed	0	690	706	661	–	415	419	971	676	196
			171	687	701	674	–	406	390	979	677	189
		Rolled FB seed	171	686	700	656	–	435	426	953	670	191
Lamminen et al. (2019)	Cows	Raw FB seed	0	729	747	671	–	696		960	–	–
			59	735	752	680	–	705		963	–	–
			117	743	760	691	–	696		965	–	–

Abbreviations: ADF, acid detergent fiber; CP, crude protein; DM, dry matter; ED, energy digestibility; EE, ether extract; N, nitrogen; NDF, neutral detergent fiber; OM, organic matter.

There are limited availability of data on the effects of FB seeds on ruminal fermentation characteristics (Table 7). The ruminal ammonia of dairy cows that were fed 171 g/kg DM of raw FB seeds increased significantly by 20.0% compared with that of dairy cows fed that were fed the SBM control diet (92 g/kg DM) (Cherif et al., 2018). Nevertheless, the pH, total volatile fatty acid (VFA) concentrations, and VFA molar proportions were similar in dairy cows that were fed with various inclusion levels of FB seeds and SBM (Cherif et al., 2018). In another study, increasing dietary inclusion levels of FB seeds in lactating cows did not affect the total VFA content and molar proportions of VFA, while the NH_3_‐N content of rumen fluid in lactating cows fed 59 or 117 g/kg DM of raw FB seeds was significantly higher compared with that of the rapeseed meal diet (Lamminen et al., 2019).

**TABLE 7:** The effect of faba bean (FB; g/kg, unless otherwise stated) seeds on ruminal fermentation characteristics

Authors	Animal	Feedstuff	FB level	pH	VFA (mM)	NH_3_‐N (mM)	Molar proportions				
							Acetate	Propionate	Butyrate	Valerate	A:P
Mariscal‐Landín et al. (2002)	Lactating cows	Raw FB TMR (g/kg DM)	0	6.26	102	6.12	0.679	0.166	0.123	0.126	4.13
			59	6.16	106	8.43	0.668	0.175	0.122	0.131	3.84
			117	6.28	100	9.37	0.670	0.169	0.126	0.130	4.00
Hejdysz et al. (2016)	Lactating cows	Raw FB TMR	0	6.09	123	9.82	0.622	0.22	0.117	0.141	2.94
			171	6.15	122	11.78	0.625	0.217	0.114	0.14	2.97
		Rolled FB TMR	171	6.2	119	11.29	0.637	0.204	0.115	0.14	3.21

Abbreviations: A:P, Acetate: Propionate; TMR, total mixed ration; VFA, volatile fatty acid.

Overall, the results indicate that FB seeds have the similar or higher nutritive value when used as a animal feed compared with the SBM and/or other leguminous seeds.

### 4.3 In vivo digestibility in nonruminants

The effects of FB seeds on the in vivo digestibility of nonruminants are summarized in Table 8. In the juvenile grass carp, increasing the inclusion of raw FB seeds up to 420 g/kg did not impair apparent digestibility coefficients of DM, CP, and ether extract (EE), while a higher inclusion of 560 g/kg adversely affected the apparent digestibility (Gan et al., 2017). In contrast, juvenile belugas fed 100 g/kg of the FB seed diet produced similar apparent digestibility coefficients for DM, CP, and EE to juvenile belugas fed wheat diets, while including FB seeds at levels higher than 150 g/kg adversely affected the belugas’ apparent digestibility (Soltanzadeh et al., 2017). Apparent digestibility coefficients of CP, EE, starch, and energy were unaffected in European seabass fed diets with various inclusion levels of extruded FB seed (Adamidou, Nengas, Alexis, et al., 2009). Moreover, apparent EE digestibility for raw FB seeds in broiler chickens ranged from 0.812 to 0.932, with high variability among cultivars (Hejdysz et al., 2016).

**TABLE 8:** Nutrient and energy digestibility, and N retention of faba bean (FB, g/kg) seed summarized from several references and different animal species

Authors	Animal	Feedstuff	FB level	Nutrient digestibility				Energy digestibility
				DM	CP	EE	Starch	
Adamidou, Nengas, Alexis, et al., 2009	European seabass	Extruded FB seed	0	‐	929	967	940	943
			150	‐	948	977	970	960
			300	‐	942	977	957	956
Hejdysz et al., 2016	Broiler chickens	Raw FB seed	400	‐	‐	872	‐	‐
		Extruded FB seed	400	‐	‐	989	‐	‐
Gan et al., 2017	Juvenile grass carp	Raw FB TMR	0	781	924	889	‐	‐
			140	783	921	887	‐	‐
			280	783	923	890	‐	‐
			420	784	923	881	‐	‐
			560	746	898	856	‐	‐
Soltanzadeh et al., 2017	Juvenile beluga	Raw FB seed	0	648	814	764	‐	‐
			50	655	813	755	‐	‐
			100	641	802	780	‐	‐
			150	617	804	713	‐	‐
			200	614	794	728	‐	‐

Abbreviations: CP, crude protein; DM, dry matter; EE, ether extract.

According to Landry et al. (2016), the apparent ileal digestibility of dietary components in male pigs fed with 629 g/kg of raw FB seeds diets was relatively high, except for NDF and ADF (Table 9). Moreover, Mariscal‐Landín et al. (2002) found that the apparent ileal digestibility of pigs fed raw FB seeds (463 g/kg) was 0.753 for DM, and 0.741 for CP, while it ranged from 0.555 to 0.862 for amino acids. Compared with lupins (*Lupinus albus* L.) diet (500 g/kg), the apparent ileal DM and OM digestibility of male broilers fed a raw FB diet (500 g/kg) was markedly higher, while the apparent ileal CP and amino acid digestibility in raw FB diets were similar to or somewhat lower than the lupin diet. In contrast, 6‐ to 32‐day‐old male broilers fed raw FB seed diets had markedly higher apparent ileal DM and OM digestibility than broilers fed the SBM control diet (170 g/kg), but apparent ileal digestibility of DM, OM, and CP were generally unaffected in broilers fed with FB seed diets with inclusion levels of 80–160 g/kg (Koivunen, Tuunainen, Rossow, et al., 2014). Moreover, Hejdysz et al. (2016) reported that apparent ileal digestibilities for broiler chickens fed a high raw FB seed diet (400 g/kg) were 0.722 for DM, 0.858 for CP, 0.760 for EE, and 0.773 for starch, respectively.

**TABLE 9:** Nutrient and energy digestibility, and N retention of faba bean (FB, g/kg) seed summarized from several references and different animal species

Authors	Animal	Feedstuff	FB level	Nutrient digestibility						
				DM	OM	CP	EE	NDF	ADF	Starch
Mariscal‐Landín et al. (2002)	Pigs	Raw FB seed	463	0.721	‐	0.708	‐	0.229	0.166	0.840
		Dehulled FB seed	417	0.753	‐	0.741	‐	‐	‐	‐
Koivunen, Tuunainen, Rossow, et al. (2014)	Male broilers	Raw FB seed	0	0.665	0.683	0.825	‐	‐	‐	‐
			80	0.696	0.721	0.831	‐	‐	‐	‐
			160	0.713	0.736	0.835	‐	‐	‐	‐
			240	0.705	0.731	0.825	‐	‐	‐	‐
Hejdysz et al. (2016)	Broiler chickens	Raw FB seed	400	0.722	‐	0.858	0.760	‐	‐	0.773
		Extruded FB seed	400	0.781	‐	0.896	0.898	‐	‐	0.970
Koivunen et al. (2016)	Broiler chickens	Raw FB seed								
	0	0.364	0.373	0.836	‐	‐	‐	‐		
Landry et al. (2016)	Male pigs	Raw FB seed	500	0.727	0.741	0.796	‐	‐	‐	‐

Abbreviations: CP, crude protein; DM, dry matter; EE, ether extract; NDF, 0neutral detergent fiber; OM, organic matter.

Overall, the aforementioned results indicate that FB seeds have a nutritive value similar to that of other legumes and/or cereals when fed to nonruminants.

## 5 IMPROVING THE UTILIZATION EFFICIENCY OF FABA BEAN SEEDS IN LIVESTOCK FEEDS

In order to maximize the nutritional value and utilization efficiency of FB seeds, it is crucial that ANFs are reduced or inactivated when they are used as ingredients in nonruminant diets (Ferruzzi et al., 2009; Khalil & Mansour, 1995). Pre‐processing of FB including dehulling, germination, soaking, and thermal treatments (i.e., cooking, autoclaving, and extrusion) was not only effective in reducing or eliminating ANFs, but also improved the intake and digestibility of nutrients (Avilés‐Gaxiola et al., 2018; Ferruzzi et al., 2009; Hejdysz et al., 2016; Masoero et al., 2005).

### 5.1 Reducing the ANFs content of faba bean seeds

A summary of the effects of processing methods on the ANFs content of FB seeds is shown in Table 10. Soaking method significantly reduced total phenolics of FB seeds by 26.7% compared with raw FB seeds (Lafarga et al., 2019) while phytic acid was generally unaffected by soaking method (Shi et al., 2018). The phytic acid content of FB seeds significantly decreased, after soaking for 4h before cooking at 95°C in water (1:5 seed:water ratio), by 29.5% of that in raw FB seeds (Shi et al., 2018). The total phenolic content of FB seeds deceased, after soaking for 24 hr before boiling in water (1:10 seed:water ratio), by 29.2% of that determined in raw FB seeds (Lafarga et al., 2019). Khalil and Mansour (1995) also reported that phytic acid, tannins, stachyose, and vicine of FB seeds decreased by 30.8%, 55.2%, 47.0%, and 35.3%, respectively, after soaking for 12 hr before cooking in tap water (3 ml/g dry seeds). Moreover, the TIA content of FB seeds significantly reduced by 50.0% and 59.6% after extrusion at 135 ± 10°C for 10 s and 52–137°C with the final pellet temperature of 121°C, respectively, while tannins were hardly affected by extrusion method (Hejdysz et al., 2016; Konieczka et al., 2020). In addition, inactivation of 41.0%, 60.0%, 40.7%, and 39.7% of the phytic acid, tannins, convicine, and vicine occurred in FB seeds after autoclaving at 121°C for 30 min, respectively (Khalil & Mansour, 1995). Contrary to the effects of a single processing method, autoclaving treatments may be optimal for reducing major ANFs.

**TABLE 10:** The effects of processing on the antinutritional factors (g/kg, unless otherwise stated) of faba bean (FB) seeds summarized from several references

Authors	Feedstuff	Tannins	TIA	Phytic acid	Convicine	Stachyose	Vicine	TP (g/100kg)
Khalil and Mansour (1995)	Raw FB seed	14.5	‐	3.9	2.7	18.1	6.8	‐
	Cooked FB seed	6.5	‐	2.7	1.8	9.6	4.4	‐
	Autoclaved FB seed	5.8	‐	2.3	1.6	14.3	4.1	‐
	Germinated FB seed	10.3	‐	1.8	1.9	0	4.9	‐
Ferruzzi et al. (2009)	Raw FB seed	6.10	‐		‐	‐	‐	‐
	Dehulled FB seed	4.69	‐		‐	‐	‐	‐
	Flaked FB seed	4.92	‐		‐	‐	‐	‐
	Cooked FB seed	2.71	‐		‐	‐	‐	‐
	Germinated FB seed	5.93	‐		‐	‐	‐	‐
Hejdysz et al. (2016)	Raw FB seed	0.06	0.6	‐	‐	‐	‐	‐
	Extruded FB seed	0.06	0.3	‐	‐	‐	‐	‐
Shi et al. (2018)	Raw FB seed	‐	‐	21.25	‐	‐	‐	‐
	Soaked FB seed	‐	‐	20.78	‐	‐	‐	‐
	Cooked FB seed	‐	‐	14.99	‐	‐	‐	‐
Lafarga et al. (2019)	Raw FB seed	‐	‐	‐	‐	‐	‐	14.7
	Soaked FB seed	‐	‐	‐	‐	‐	‐	10.78
	Cooked FB seed	‐	‐	‐	‐	‐	‐	10.41
Konieczka et al. (2020)	Raw FB seed	0.046	0.570	‐	‐	‐	‐	‐
	Extruded FB seed	0.046	0.230	‐	‐	‐	‐	‐

Abbreviations: TIA, trypsin inhibitor activity; TP, total phenolic.

Relative to the preprocessing methods used, selective breeding may be the most effective method in reducing or removing the ANFs of FB seeds (Warsame et al., 2018). The tannin content of three FB varieties with low tannin content (Snowbird, CDC Snowdrop, and CDC 219–16) were only average 11.9% of three varieties with normal tannin content (CDC Fatima, 346–10, and CDC SSNS‐1) (Espinosa et al., 2020). The use of a robust molecular marker is available for marker‐assisted breeding to reduce the vicine and convicine contents of FB seeds (Khazaei, Purves, et al., 2019; Robinson et al., 2019). The development of sequences that had amplified marker regions could be applied to track the two genes (zt1 and zt2) as molecular markers for speeding up the breeding of new FB varieties with low tannins (Zanotto et al., 2019), while gene zv has been incorporated into the FB plant for low or zero vicine and convicine content (Olson & Bowness, 2016). A gene labeling method has been used for facilitating indirect selection of FB seed quality traits, including a zero tannin and low vicine and convicine content (Alghamdi et al., 2012). Signor et al. (2017) reported that 52 genes present in the pathways resulting in globulin accumulation had potential in selection for higher seed nutritive value. In addition, Prabhu and Rajeswari (2018) reported that γ‐aminobutyric acid and diamine oxidase also modified the ANFs of legumes.

Overall, the literature suggests that various processing methods markedly inactivate or reduce the ANFs of FB seeds; this is especially true for heat treatments, which have been highly effective in reducing ANFs.

### 5.2 Improving the nutritive value of faba bean seeds

The proximate nutritional composition and essential amino acid and mineral contents (except for potassium and magnesium) of FB seed only change slightly when subjected to cooking, autoclaving, flaking, and germination (Table 11) (Ferruzzi et al., 2009; Khalil & Mansour, 1995; Schwediauer et al., 2018). The extrusion treatment caused a marked reduction in the NDF, EE, and resistant starch contents of FB seeds, while it did not affect other chemical parameters or the amino acid profile of the FB seed (Hejdysz et al., 2016; Lestingi et al., 2015; Masoero et al., 2005).

**TABLE 11:** The effects of processing on the nutritive composition (g/kg DM) and in vitro digestibility of faba bean (FB) seeds summarized from several references

Authors	Feedstuff	Nutritive composition								In vitro digestibility			PER
		CP	EE	CF	NDF	ADF	ADL	Starch	Sugar	OM	NDF	CP	
Khalil and Mansour (1995)	Raw FB seed	292	11	‐	‐	‐	‐	‐	‐	‐	‐	0.646	2.40
	Cooked FB seed	290	10	‐	‐	‐	‐	‐	‐	‐	‐	0.712	2.70
	Autoclaved FB seed	275	10	‐	‐	‐	‐	‐	‐	‐	‐	0.737	2.60
	Germinated FB seed	305	9	‐	‐	‐	‐	‐	‐	‐	‐	0.722	2.60
Masoero et al. (2005)	Raw FB seed	293	18.2		313	129	‐	371	45.6	‐	‐	‐	‐
	Extruded FB seed	292	20.1		230	147	‐	382	66.0	‐	‐	‐	‐
Ferruzzi et al. (2009)	Raw FB seed	295	12.6	‐	245	135	19.1	‐	‐	0.914	0.518	‐	‐
	Dehulled FB seed	338	12.2	‐	123	23.5	7.2	‐	‐	0.993	0.903	‐	‐
	Flaked FB seed	297	12.9	‐	213	129	17.7	‐	‐	0.925	0.554	‐	‐
	Cooked FB seed	290	12.8	‐	241	174	15.9	‐	‐	0.895	0.487	‐	‐
	Germinated FB seed	302	19.3	‐	242	112	19.9	‐	‐	0.904	0.391	‐	‐
Koivunen, Tuunainen, Valkonen, et al. (2014)	Raw FB seed	302	22.7	93.9	‐	‐	‐	‐	‐	‐	‐	‐	‐
	Expanded FB seed	285	21.5	95.5	‐	‐	‐	‐	‐	‐	‐	‐	‐
Lestingi et al. (2015)	Raw FB seed	293	17.8	‐	313	129	‐	370	‐	‐	‐	‐	‐
	Extruded FB seed	292	19.8	‐	229	147	‐	382	‐	‐	‐	‐	‐
Hejdysz et al. (2016)	Raw FB seed	312	10.0	‐	213	124	‐	417	‐	‐	‐	‐	‐
	Extruded FB seed	310	6.00	‐	132	119	‐	411	‐	‐	‐	‐	‐
Schwediauer et al. (2018)	Raw FB seed	317	15.0	81.0	‐	‐	‐	‐	‐	‐	‐	‐	‐
	Germinated FB seed	321	15.0	85.0	‐	‐	‐	‐	‐	‐	‐	‐	‐

Abbreviations: ADF, acid detergent fiber; ADL, acid detergent lignin; CF, crude fiber; CP, crude protein; EE, ether extract; PER, protein efficiency ratio; NDF, neutral detergent fiber; OM, organic matter.

Cooking, autoclaving, dehulling, flaking, extrusion, and germination changed the in vitro digestibility of the nutrients in FB seeds. In vitro CP digestibility of FB seeds significantly increased by 10.2%, 14.1%, and 11.8% after cooking in tap water (3 ml/g dry seeds), autoclaving at 121°C for 30 min, and germinating at room temperature for 3 days, respectively, because of the reduction or inactivation of ANFs (Khalil & Mansour, 1995). However, cooking, autoclaving, and germinating improved PER slightly (Khalil & Mansour, 1995). The apparent digestibility of EE and ME of FB seeds increased significantly by 8.17% and 4.43%, respectively, after extrusion at 135°C for 10 s with a moisture content of 22% (Hejdysz et al., 2016). Dehulling and flaking the FB seeds significantly increased their in vitro OM digestibility (by 8.64% and 1.20%, respectively) and in vitro NDF digestibility (by 74.3% and 6.95%, respectively); however, the cooking and germination treatments did not increase this digestibility and even reduce the digestibility in some cases (Ferruzzi et al., 2009). Moreover, extrusion treatment significantly improved the apparent EE digestibility and apparent ileal digestibility of DM, CP, and EE of FB seeds by 13.4%, 8.17%, 4.43%, and 18.2%, respectively (Hejdysz et al., 2016).

Traditional breeding approaches coupled with gene transfer studies and functional genomics would be useful for the breeding of FB lines and the development of new FB cultivars with novel protein profiles or properties with added value (Gutierrez et al., 2007; Robinson et al., 2019). Avila et al. (2007) also reported that codominant markers could promote the breeding process of FB and be useful for the quality control of FB seeds.

Overall, the literature suggests that the nutritional value of FB seeds is improved by various processing methods, especially extrusion treatment, through the inactivation or reduction in the ANFs.

## 6 ANIMAL FEED STUDIES USING FABA BEAN SEEDS

### 6.1 Ruminants

#### 6.1.1 Lactating ruminants

In the Liponi et al. (2007) study, raw FB seeds replaced SBM at inclusions of 320 g/kg in the concentrate of lactating Massese ewes without affecting the milk yield, or milk fat, protein, and lactose content (Table 12), which is consistent with Mordenti et al. (2007) who found that Holstein dairy cows fed a concentrate of 345 g/kg DM FB seeds had a similar productive performance to cows fed with an SBM concentrate (150 g/kg DM). Puhakka et al. (2016) evaluated the effects of partially or completely substituting FB seeds for rapeseed meal on the milk production and composition of Finnish Ayrshire cows. The rapeseed meal and FB seeds were included in the concentrate that were fed to the cows in different ratios (129:0, 64.6:75.1, 0:150, 152:175, and 0:350), and no differences were found in average milk fat (4.20%) and lactose (4.59%) contents (Puhakka et al., 2016). However, higher inclusion levels of 350 g/kg DM somewhat reduced the milk yield, although no differences in DM intake and milk yield were found at FB inclusions ≤345 g/kg DM of concentrate (Puhakka et al., 2016).

**TABLE 12:** The effect of faba bean (FB; g/kg DM, unless otherwise stated) seed on performance of lactating ruminants summarized from several references and different animal species

Authors	Animal	Feedstuff	FB level	DM (kg/day)	Milk yield (L/day)	FE (milk/DMI)	Fat (%)	CP (%)	Lactose (%)
Liponi et al. (2007)	Ewes	Raw FB concentrate (g/kg)	0	‐	0.784	‐	6.58	6.39	4.25
			320	‐	0.730	‐	6.76	6.54	4.57
Morales et al. (2008)	Ewes	Raw FB TMR (g/kg)	1.51	‐	‐	5.20	2.88	4.50	
			210	1.51	‐	‐	5.25	3.12	4.23
Tufarelli et al. (2012)	Cows	Raw FB concentrate	0	23.1	27.2	‐	3.63	3.16	5.01
			345	22.9	27.1	‐	3.53	3.14	5.07
Puhakka et al. (2016)	Cows	Raw FB concentrate	0	20.3	30.8	‐	4.19	3.39	4.59
			75.1	20.1	30.3	‐	4.20	3.29	4.60
			150	19.4	29.5	‐	4.23	3.27	4.58
			175	20.0	31.1	‐	4.16	3.28	4.58
			350	18.7	28.9	‐	4.23	3.22	4.60
Cherif et al. (2018)	Cows	Raw FB TMR	0	25.7	36.5	1.43	3.92	3.42	4.50
			171	25.6	35.8	1.40	3.90	3.40	4.52
		Rolled FB TMR	171	26.0	36.0	1.39	3.90	3.39	4.49

Abbreviations: CP, crude protein; DMI, dry matter intake; FE, feed efficiency; TMR, total mixed ration.

The total replacement of raw bitter vetch (*Vicia ervilia*) seeds with raw FB seeds on milk yield and composition of dairy goats produced no differences in milk yield, or milk fat, protein, and lactose contents (Morales et al., 2008). In another study, substituting a raw or rolled FB seed (at a level of 171 g/kg DM diet) for SBM (at a level of 9.2 g/kg DM diet) did not affect the milk yield, or milk fat, protein, and lactose content of lactating Holstein cows (Cherif et al., 2018).

#### 6.1.2 Growing ruminants

Using male Comisana lambs, Bonanno et al. (2012) evaluated the nutritive value of raw FB seeds in diets where raw FB seeds replaced SBM in the concentrate in proportions of 250:0 and 0:758 g/kg for SBM and FB seeds, respectively (Table 13). They reported that no differences were found in average daily feed intake (ADFI), average daily gain (ADG), feed conversion rate (FCR), or carcass yield (Bonanno et al., 2012). Furthermore, male Fabrianese lambs fed a concentrate with 242 g/kg raw FB seeds had a similar productive performance to lambs fed a SBM concentrate (160 g/kg) (Polidori et al., 2018).

**TABLE 13:** Effect of faba bean (FB; g/kg) seed on the performance of growing ruminants summarized from several references

Authors	Lambs	Feedstuff	FB level	ADFI (kg/day)	ADG (kg/day)	FCR (ADFI/ADG)	Carcass yield (% BW)
Lanza et al. (1999)	Male lambs	Raw FB TMR	0	‐	0.233	‐	46.1
			538	‐	0.219	‐	46.1
Bonanno et al. (2012)	Male lambs	Raw FB concentrate	0	0.800	0.186	4.68	45.3
			758	0.826	0.178	4.82	45.7
Lestingi et al. (2015)	Male lambs	Raw FB TMR	0	‐	0.130	6.38	50.4
			150	‐	0.170	5.17	47.4
			300	‐	0.180	4.97	46.8
Polidori et al. (2018)	Male lambs	Raw FB concentrate	0	1.13	0.199	5.69	55.6
			242	1.14	0.186	6.13	54.3
Ragni et al. (2018)	Heifers	Raw FB TMR	0	8.60	1.21	7.17	‐
			280	7.82	1.18	6.71	‐

Abbreviations: ADFI, average daily feed intake; ADG, average daily gain; BW, body weight; FCR, feed conversion ratio; TMR, total mixed ration.

In an 8‐week experiment, male Barbaresca lambs that were fed either a SBM diet (206 g/kg) or a FB seed diet (538 g/kg) had similar final body weight (BW, 27.1 kg) and ADG (0.226 kg/day) [60]. In another study, Lestingi et al. (2015) studied the effects of partially and completely substituting raw FB seeds for lupin on the productive performance of growing lambs. The lambs were fed diets containing lupin seed to FB seed ratios of 250:0 g/kg (control), 150:150 g/kg, and 0:300 g/kg, and increasing the raw FB seed content in the diet accelerated the productive performance. For Charolais heifers, animals fed a diet of 280 g/kg FB seeds had similar final BW, ADG, and ADFI to heifers fed the SBM control diet (140 g/kg); however, the FB seed diet has significantly less FCR compared with the SBM diet (Ragni et al., 2018).

In addition, Fabrianese entire male lambs slaughtered at 145 days of age did not differ in terms of their slaughter performance or the physical and chemical traits of their *longissimus dorsi* muscle when fed with a SBM diet (160 g/kg of diet) or a diet containing 242 g/kg of raw FB seeds (Polidori et al., 2018). Similarly, Bonanno et al. (2012) also found that slaughter parameters, physical and chemical characteristics of the *longissimus dorsi* muscle, and perirenal fat color of lambs slaughtered at ~129 days of age were not affected when raw FB seeds were added to the concentrate, even at 758 g/kg. Gentile di Puglia male lambs slaughtered at 98 days of age had similar carcass traits and nutritional composition of leg and loin tissue among dietary treatments containing raw FB seeds up to 300 g/kg (Lestingi et al., 2015). Similarly, diets supplemented with 538 g/kg raw FB seeds had no effect on carcass yield and fat yield, lean meat yield, or the physical, chemical, and sensory traits of their *longissimus dorsi* muscle compared with the SBM control diet (206 g/kg) (Lanza et al., 1999). Charolais heifers slaughtered at approximately 119 kg BW did not differ in slaughtering parameters and dissection parameters of the pelvic limb and lumbar region as well as physical and chemical characteristics of meat from *longissimus lumborum* muscle (Ragni et al., 2018).

Overall, the literature suggests that substituting FB seeds for SBM or other legume seeds results in equal or somewhat increased growth as well as increased milk yield and composition in ruminants.

### 6.2 Pigs

Using female pigs, O’Doherty and McKeon (2001) reported on the nutritive value of raw and extruded FB seeds in their diets (Table 14). The pigs were fed diets that included 0, 125, 250, and 375 g/kg of raw FB seeds and 0, 250, and 375 g/kg of extruded FB seeds, respectively. Increasing the FB content in the diet did not affect the FCR and carcass characteristics, while no differences were observed in ADFI and ADG in the raw FB seed inclusion groups; however, ADFI and ADG declined linearly with increasing extruded FB seed in the diet. In addition, Gunawardena et al. (2010) found that substituting raw or dehulled FB seeds (160 g/kg) for soy protein concentrate‐corn gluten meal‐menhaden meal diets (160 g/kg) did not affect the final BW, ADFI, ADG, and FCR of weaned pigs compared with control diet (without the FB seeds). Moreover, Schwediauer et al. (2018) reported that raw or germinated FB seeds (160 g/kg) could partially replace peas at inclusion levels of 160 g/kg in the diet without affecting the final BW, ADFI, ADG, and FCR of weaner piglets, while germinated FB seeds at a higher inclusion level of 240 g/kg in the diet could adversely affect the piglets’ productive performance (Schwediauer et al., 2018).

**TABLE 14:** Effect of faba bean (FB; g/kg) seed on the performance of pigs summarized from several references

Authors	Lambs	Feedstuff	FB level	ADFI (kg/day)	ADG (kg/day)	FCR (kg ADFI/kg ADG)	Carcass yield (% BW)
O’Doherty and McKeon (2001)	Female pigs	Raw FB TMR	0	2.25	0.89	2.50	72.63
			125	2.21	0.87	2.53	73.59
			250	2.16	0.85	2.53	73.71
			375	2.21	0.85	2.59	74.42
		Extruded FB TMR	250	2.13	0.84	2.49	74.89
			375	2.10	0.82	2.55	75.67
Gunawardena et al. (2010)	Pigs	Raw FB TMR	0	0.663	0.49	1.36	‐
			160	0.649	0.48	1.34	‐
		Dehulled FB TMR	160	0.653	0.48	1.35	‐
Smith et al. (2013)	Growing pigs	Raw FB TMR	0	1.86	0.82	2.27	‐
			75	1.98	0.85	2.33	‐
			150	2.00	0.86	2.33	‐
			225	2.07	0.90	2.27	‐
			300	2.01	0.91	2.22	‐
	Finisher pigs		0	2.70	1.08	2.50	‐
			75	2.53	1.02	2.56	‐
			150	2.68	1.01	2.70	‐
			225	2.59	0.98	2.56	‐
			300	2.63	1.03	2.56	‐
Schwediauer et al. (2018)	Weaner piglets	Raw FB TMR	0	0.74	0.39	1.99	‐
			160	0.73	0.40	1.93	‐
		Germinated FB TMR	160	0.75	0.38	2.10	‐
			240	0.73	0.34	2.13	‐
Grabež et al. (2020)	Pigs	Raw FB TMR	0	2.24	1.09	2.06	64.62
			161	2.27	1.08	2.12	64.79

Abbreviations: ADFI, average daily feed intake; ADG, average daily gain; BW, body weight; FCR, feed conversion ratio; TMR, total mixed ration.

In addition, Grabež et al. (2020) showed that Norwegian crossbred pigs that were fed a SBM diet (143 g/kg) or a FB seed diet (161 g/kg) had similar growth performances, carcass characteristics, meat quality, and mostly similar fatty acid composition of *longissimus thoracis* muscle. Smith et al. (2013) studied the effects of partially and completely substituting raw FB seeds for SBM on the growth performance and carcass quality of growing/finisher pigs. SBM and FB seeds were fed to pigs in proportions of 140:0, 105:75, 70:150, 35:225, and 0:300 g/kg, and no differences were found in the FB seed inclusion groups in terms of the ADFI, ADG, FCR, carcass quality, or backfat skatole content (Smith et al., 2013).

Overall, the literature suggests that substituting SBM or peas for FB seeds in pig feedstuffs does not affect their growth performance, carcass characteristics, or meat quality.

### 6.3 Poultry

#### 6.3.1 Laying hens

Using NovoGen White hens, Moujahed et al. (2020) evaluated the nutritive value of raw FB seeds in diets where FB seeds replaced SBM in proportions of 200:0, 165:50, and 135:100 g/kg, respectively. Laying hens fed FB seeds had significantly lower feed intake (FI), egg production (EP), and egg weight (EW) compared with the SBM control diet, while FB seeds at higher inclusion level of 100 g/kg in the diet positive affected the egg shape index and yolk color (Moujahed et al., 2020). Laudadio and Tufarelli (2010) showed that laying hens fed with a 240 g/kg diet of FB seeds had a similar productive performance to those fed the SBM control diet (150 g/kg). In contrast, layers that were fed diets with 298 g/kg of raw FB seeds had similar final BW, FI, EW, and eggshell strength as layers fed SBM diets (72.0 g/kg), while the EP of the former was reduced by 12.8% compared with that of the latter (Laudadio & Tufarelli, 2010). Similarly, Abd el‐Hack et al. (2017) showed that raw FB seeds could partially replace SBM at a level of 110 g/kg without affecting the FI, EP, egg mass (EM), EW, feed efficiency (FE), or egg quality criteria of Hisex Brown laying hens; however, higher inclusion levels of 165 or 220 g/kg adversely affected the hens’ egg production and quality.

A study by Olaboro et al. (1980) studied the effect of substituting FB seeds (400 g/kg) processed in three different ways (dehulled, autoclaved at 121°C for 30 min, and dehulled and autoclaved at 121°C for 30 min) for raw FB seeds on the egg‐laying performance of layers (Table 15). The authors found no differences among the processed FB seed groups in terms of their average FI (105.3 g/day), EP (0.816 eggs/hen/day), EM (46.4 g/hen/day), EW (56.8 g), and FE (2.23). Koivnen, Tuunainen, Valkonen et al. (2014a) studied the nutritive value of raw and expanded FB seeds (0, 50, and 100 g/kg) in the diets of laying hens. Increasing FB seed content in the diet did not affect the FI and EP, and there were no differences between raw and expanded FB groups, while the EM declined and FE increased in both groups (Koivunen, Tuunainen, Valkonen, et al., 2014).

**TABLE 15:** Effect of faba bean (FB; g/kg) seed on the performance of ​laying hens summarized from several references

Authors	Animal	Feedstuff	FB level	FI (g/day)	EP (eggs/hen/day)	EM (g/hen/day)	EW (g)	FE (g FI/g EM)
Olaboro et al. (1980)	Laying hens	Raw FB TMR	400	106.8	0.795	45.4	57.1	2.40
		Autoclaved FB TMR	400	109.1	0.828	46.9	56.6	2.30
		Dehulled FB TMR	364	104.2	0.827	47.5	57.3	2.20
		Autoclaved dehulled FB TMR	364	101.0	0.814	45.6	56.0	2.20
Laudadio and Tufarelli (2010)	Laying hens	Raw FB TMR	0	107.1	0.8067	‐	55.7	1.98
			240	105.5	0.7811	‐	54.1	2.02
			298	116.0	0.689	‐	55.2	3.05
Koivunen, Tuunainen, Valkonen, et al. (2014)	Laying hens	Raw FB TMR	0	114.5	0.900	59.5	66.1	1.93
			50	114.3	0.914	59.0	64.6	1.94
			100	122.4	0.880	57.2	65.1	2.14
		Expanded FB TMR	50	116.9	0.909	59.7	65.7	1.97
			100	116.6	0.909	58.4	64.3	2.00
Abd El‐Hack et al. (2017)	Laying hens	Raw FB TMR	0	106.5	0.907	62.9	69.2	1.70
			55	106.9	0.912	63.9	69.8	1.70
			110	107.7	0.910	62.8	68.8	1.72
			165	97.8	0.795	51.9	65.1	1.90
			220	86.1	0.715	45.2	63.2	1.92
Moujahed et al. (2020)	Laying hens	Raw FB TMR	0	108.5	0.871	‐	61.0	2.17
			50	107.05	0.816	‐	60.3	2.18
			100	106.9	0.832	‐	60.0	2.24

Abbreviations: EM, egg mass; EP, egg production; EW, egg weight; FE, feed efficiency; FI, feed intake; TMR, total mixed ration.

#### 6.3.2 Broiler chickens

Using male Ross 508 broilers, FB seeds replaced SBM in the diets in proportions of 186:0, 153:80, 119:160, and 86:240 g/kg (Table 16; Koivunen, Tuunainen, Valkonen, et al., 2014). No differences were observed in the growth performance of the lower FB seed inclusion level group and the SBM group; however, the highest FB seed inclusion group had a 10.9% lower daily feed consumption (DFC) and 5.59% lower BW gain than the SBM group (Koivunen, Tuunainen, Valkonen, et al., 2014). In contrast, DFC, meat traits, content of muscles, and fat, as well as major physicochemical parameters of breast muscles and leg muscles for male ROSS 308 chicks were not affected in SBM substitutions of 250:0 g/kg (control) versus 0:250 g/kg (Biesek et al., 2020). However, broilers fed FB seeds had significantly 29.1% higher FCR and 18.9% lower ADG than the SBM control diet (Biesek et al., 2020). Increasing the dehulled FB seed ratio up to 250 g/kg in broiler chickens’ diets did not affect the growth performance of broilers [38], which can be attributed to the improved nutrient composition and in vitro digestibility of nutrients as well as the reduced tannin content of the dehulled FB seeds (Ferruzzi et al., 2009). Furthermore, in a 4‐week experiment, female Ross 308 broiler chickens fed either a raw or extruded (300 g/kg) FB seed diet had a similar DFC (112 g), ADG (78.2 g/day), and FCR (1.44) (Konieczka et al., 2020).

**TABLE 16:** Effect of faba bean (FB; g/kg) seed on the performance of broilers summarized from several references

Authors	Animal	Feedstuff	FB level	DFC (g/day)	BW gain (g/day)	FCR (g DFC/g BW gain)
Gous (2011)	Broilers (7–21 days of age)	Dehulled FB TMR	0	55.9	35.4	0.633
			50	57.4	36.6	0.636
			100	57.0	35.7	0.624
			150	55.8	34.6	0.619
			200	58.0	36.2	0.622
			250	56.6	34.6	0.608
Koivunen et al. (2016)	Broilers (6–32 days of age)	Raw FB TMR	0	110	69.7	1.63
			80	104	69.0	1.58
			160	103	69.4	1.56
			240	98	65.8	1.55
Biesek et al. (2020)	Broilers (0–42 days of age)	Raw FB TMR	0	94.5	61.9	1.51
			250	97.5	50.2	1.95
Konieczka et al. (2020)	Broilers (8–35 days of age)	Raw FB TMR	300	113	77.5	1.46
		Extruded FB TMR	300	111	78.9	1.41

Abbreviations: DFC: daily feed consumption; BW: body weight; FCR: feed conversion ratio; TMR: total mixed ration.

Overall, the literature suggests that adding FB seeds to layer or broiler diets does not affect the EP of layers or the EP and growth performance of broilers.

### 6.4 Fish

In a study by Adamidou, Nengas, Henry, et al. (2009), in which European seabass were fed diets with the complete substitution of 165 g/kg extruded FB or extruded field pea seeds for extruded wheat (170 g/kg), there were no differences in the FB or field pea groups in terms of final BW, ADFI, ADG, FCR, or proximate composition of the carcass (Table 17). Adamidou et al. (2011) showed that the productive performance and major carcass proximate composition of Gilthead seabream were not affected by the inclusion of extruded FB seeds (175 g/kg) that partially substituted wheat, corn gluten, and wheat gluten in the diets.

**TABLE 17:** The effect of faba bean (FB; g/kg as‐fed basis) seed on performance of fish summarized from several references

Authors	Animal	Feedstuff	FB level	ADFI (g/day/fish)	Initial BW (g)	Final BW (g)	ADG (g/day^/^fish)	FCR (ADFI/ADG)	PER
Adamidou, Nengas, Henry, et al. (2009)	European seabass	Extruded FB TMR	0	‐	102.4	250.5	1.51	1.34	‐
			165	‐	100.1	264.6	1.68	1.31	‐
Azaza et al. (2009)	Juvenile nile tilapia	Raw FB TMR	0	2.22	17.3	116.3	1.32	1.56	2.34
			120	2.20	17.2	117.9	1.34	1.62	2.25
			240	2.17	17.3	116.0	1.31	1.58	2.30
			360	1.96	17.3	100.6	1.11	1.79	2.04
Adamidou et al. (2011)	Gilthead seabream	Extruded FB TMR	0	2.21	95.1	216.2	1.40	1.58	‐
			175	2.07	89.9	188.2	1.20	1.72	‐
Gan et al. (2017)	Juvenile grass carp	Raw FB TMR	0	‐	3.39	56.08	0.941	1.09	2.78
			140	‐	3.38	56.99	0.957	1.06	2.83
			280	‐	3.38	57.31	0.963	1.08	2.76
			420	‐	3.39	58.88	0.991	1.06	2.76
			560	‐	3.39	52.48	0.877	1.23	2.38
Soltanzadeh et al. (2017)	Juvenile beluga	Raw FB TMR	0	‐	82.89	257.8	3.12	0.70	0.295
			50	‐	82.91	251.6	3.01	0.73	0.302
			100	‐	82.58	248.0	2.95	0.75	0.302
			150	‐	81.91	242.2	2.86	0.76	0.314
			200	‐	81.62	239.2	2.81	0.79	0.318
			250	‐	82.33	238.1	2.78	0.82	0.327

Abbreviations: ADFI, average daily feed intake; ADG, average daily gain; BW, body weight; FCR, feed conversion ratio; PER, Protein efficiency ratio; TMR, total mixed ration.

Additionally, Azaza et al. (2009) evaluated the nutritive value of FB seeds in the diets of juvenile Nile tilapia fed dehulled SBM and raw FB seeds in ratios of 450:0, 350:120, 250:240, and 150:360 g/kg for SBM and FB seeds, respectively. No differences were detected in terms of the final BW, ADFI, ADG, and PER between the group with the lower FB seed level and the SBM group; however, the Nile tilapia with the highest FB seed inclusion had a 13.5% lower final BW, 11.7% lower ADFI, 15.9% lower ADG, and 12.8% lower PER than the fish fed dehulled SBM (Azaza et al., 2009). Similarly, the inclusion of 100 g/kg of raw FB seeds in the diets of juvenile belugas did not affect their growth performance, while a higher inclusion level of 150, 200, or 250 g/kg of diets negatively affected growth performance (Soltanzadeh et al., 2017). Raw FB seeds could be used as partial substitutes for SBM at lower inclusion levels (<420 g/kg) without affecting the ADFI, final BW, ADG, and FCR of juvenile grass carp, while a higher inclusion level (560 g/kg) negatively affected their growth performance (Gan et al., 2017). These results suggest that fish might be susceptible to the adverse effects of the ANFs found in diets with more raw FB seeds.

Overall, the literature suggests that substituting low amounts of raw FB seeds for SBM and cereal grains in fish diets do not affect the growth performance of fish.

## 7 CONCLUSIONS

FB seeds are high in protein and energy and are used as an alternative feedstuff in livestock production. To support higher growth and/or productive performance of animals, raw FB seeds can be generally included in cow concentrate and lamb diets at appropriate levels as 175 and 300 g/kg, respectively, while raw FB seeds can be used in pig, layer, broiler (6–32 days of age), and fish diets at appropriate levels of up to 300, 110, 160, and 420 g/kg, respectively. The inclusion of higher levels of FB seeds in pig, poultry, and fish diets is possible after the ANFs have either been eradicated or reduced with the use of preprocessing treatments to improve the nutritional value of the seeds. Of the preprocessing treatments, extrusion treatment facilitates the inclusion of higher FB seed levels in the diets of nonruminants without any adverse effects on their performance.

## CONFLICT OF INTEREST

The authors declare that they have no competing interests.

## AUTHOR CONTRIBUTION

**Zhu Meng:** Software (equal); Writing‐original draft (equal); Writing‐review & editing (equal). **Qingqing Liu:** Data curation (equal); Investigation (equal); Methodology (equal); Writing‐original draft (equal); Writing‐review & editing (equal). **Yan Zhang:** Data curation (equal); Software (equal). **Jiahong Chen:** Data curation (equal); Investigation (equal); Software (equal). **Zhipeng Sun:** Data curation (equal); Investigation (equal); Software (equal). **Chunhuan Ren:** Data curation (equal); Funding acquisition (equal). **Zijun Zhang:** Funding acquisition (equal); Writing‐review & editing (equal). **Xiao Cheng:** Data curation (equal); Writing‐original draft (equal). **Yafeng Huang:** Data curation (equal); Formal analysis (equal); Software (equal); Writing‐original draft (equal); Writing‐review & editing (equal).

## ETHICAL APPROVAL

No ethical approval was required, as this is a review article with no original research data.
